# Gender-Based Deep Learning Firefly Optimization Method for Test Data Generation

This article has been retracted.

**DOI:** 10.1155/2021/8056225

**Published:** 2021-05-28

**Authors:** Wenning Zhang, Chongyang Jiao, Qinglei Zhou, Yang Liu, Ting Xu

**Affiliations:** ^1^State Key Laboratory of Mathematical Engineering and Advanced Computing, Zhengzhou, Henan 450000, China; ^2^Software College, Zhongyuan University of Technology, Zhengzhou, Henan 450000, China; ^3^School of Information Engineering, Zhengzhou University, Zhengzhou, Henan 450000, China; ^4^The Jackson Laboratory for Genomic Medicine, Farmington 06032, CT, USA

## Abstract

Software testing is a widespread validation means of software quality assurance in industry. Intelligent optimization algorithms have been proved to be an effective way of automatic test data generation. Firefly algorithm has received extensive attention and been widely used to solve optimization problems because of less parameters and simple implement. To overcome slow convergence rate and low accuracy of the firefly algorithm, a novel firefly algorithm with deep learning is proposed to generate structural test data. Initially, the population is divided into male subgroup and female subgroup. Following the randomly attracted model, each male firefly will be attracted by another randomly selected female firefly to focus on global search in whole space. Each female firefly implements local search under the leadership of the general center firefly, constructed based on historical experience with deep learning. At the final period of searching, chaos search is conducted near the best firefly to improve search accuracy. Simulation results show that the proposed algorithm can achieve better performance in terms of success coverage rate, coverage time, and diversity of solutions.

## 1. Introduction

Software testing is a labor-intensive and significant measure of software quality accounting for more than 40% of total cost [1]. Automating the process of test data generation to search feasible test cases to satisfy given testing criteria (e.g., branch coverage) can reduce testing cost thus the overall cost, increasing the software quality [2]. Automatic test data generation for path coverage-based optimization is one of the most basic and critical domains with considerable research interest. Its purpose is to generate test data to execute each feasible path of the program at least once [3].

Inspired by human intelligence and natural phenomena of biological groups, more and more metaheuristic algorithms are proposed to solve diverse optimization applications and show their unique advantages. Since many typical questions in software engineering can be formulated as optimization question, search-based software engineering (SBSE) has been widely applied during the whole software life cycle, such as requirement and project management. As a sub area of SBSE, search-based software testing (SBST) has received the most widespread study and been proved to be an effective approach to generate structural test case [4, 5]. Metaheuristic algorithms that have been used in test case generation include genetic algorithms, particle swarm optimization, firefly algorithm, artificial bee colony, cuckoo search algorithm, ant colony optimization, and others [2].

Through the simulation and simplification of the behavior of fireflies, Yang [6] developed the firefly algorithm (FA) according to the flashing patterns of fireflies. As one of the stochastic, swarm intelligence methods, it has been received extensive attention and successfully applied to various applications because of its efficiency and simplicity [7, 8]. However, FA shows some drawbacks such as low accuracy and falling into local optima. To overcome the aforementioned limitations, we intend to propose a gender difference-based firefly algorithm with deep learning to generate structural test case.

This paper proposed an effective metaheuristic firefly search algorithm for structural test data generation, which is the most widely studied of all the applications of search-based techniques to the test data generation problem. The main work can be concluded as follows: first, a solution to generate test case used FA is constructed; second, a new algorithm by combining random attraction model, deep learning, and chaotic search is formulated to balance the global and local search ability; third, the implementation and its analysis on public benchmark programs are discussed in detail.

## 2. Background

### 2.1. Firefly Algorithm

FA is a metaheuristic algorithm motivated by the idealized biological behavior and information interaction strategy of fireflies. The less bright firefly will be attracted and moved towards the brighter one. Generally, attractiveness between two fireflies is proportional to the brightness and inversely proportional to the distance [6]. In the process of evolution, fireflies will gradually focus on the brightest fireflies, which are target solutions. In search space of optimization problems, especially maximization problems, the firefly brightness can simply be computed to the encoded fitness function value, and each firefly represents a candidate solution of optimization problem.

Assuming there are *N* fireflies in *D*-dimensional space, the any two *i*th/*j*th firefly can be represented as *x*_*i*_=(*x*_*i*1_, *x*_*i*2_,…, *x*_*iD*_),  *i*=1,2,…, *N* and *x*_*j*_=(*x*_*j*1_, *x*_*j*2_,…, *x*_*ij*_),  *j*=1,2,…, *N*, respectively. The mathematical description of FA can be described as follows [9].

Each firefly should be initialized as follows:

(1) $$\begin{array}{c} x_{ij}=\mathrm{rand}\left(\right)*\left(U-L\right), \end{array}$$

where rand() is randomization function generating numbers between 0 and 1 and *U* and *L* are upper bound and lower bound of the input space.

The distance between firefly *i* at *x*_*i*_ and firefly *j* at *x*_*j*_ can be defined as follows:

(2) $$\begin{array}{c} r_{ij}=\left\|x_{i}-x_{j}\right\|=\sqrt{\sum_{d=1}^{D}{\left(x_{id}-x_{jd}\right)}^{2}}, \end{array}$$

where *x*_*id*_ is the *d*th spatial coordinate of the *i*th firefly and *x*_*jd*_ is the *d*th spatial coordinate of the *j*th firefly.

To reduce complexity of optimization, especially in the simplest maximum problems, the attractiveness of firefly *i* can be formulated as *I*(*i*), determined by its brightness associated with the fitness function value. Supposing firefly *j* is brighter than firefly *i*, the firefly *i* will be attracted and moved to firefly *j*. However, the brightness seen by firefly *i* will decrease with the distance because of the media light absorption. Then, the attractiveness will change according to the degree of absorption. Considering the absorption and inverse square law, the light intensity can be defined as in (3) and the relative attractiveness can be defined as in (4).

(3) $$\begin{array}{c} I_{ij}\left(r_{ij}\right)=I_{i}e^{-\gamma r_{ij}^{2}}, \end{array}$$

(4) $$\begin{array}{c} \beta_{ij}\left(r_{ij}\right)=\beta_{0}e^{-\gamma r_{ij}^{2}}, \end{array}$$

where *I*_*i*_ is attractiveness of firefly *i* according to the encoded fitness function, *γ* is a given light absorption coefficient, and *β*_0_ is the initial attractiveness when *r* = 0.

The movement of firefly *i* attracted by firefly *j* is defined as follows:

(5) $$\begin{array}{c} x_{id}\left(t+1\right)=x_{id}\left(t\right)+\beta \left(x_{jd}\left(t\right)-x_{id}\left(t\right)\right)+\alpha_{i}\left(t\right)\varepsilon , \end{array}$$

where the second part is the attractiveness between two fireflies and the third part is the random walk.

### 2.2. Related Research

There are many complex optimization problems in many fields, which cannot be solved by traditional optimization approaches. With the deep learning from society and nature, the last decades has seen the emergence of many new meta heuristic search algorithms, such as genetic algorithm (GA), hill climbing algorithm (HCA), particle swarm optimization (PSO), cuckoo search algorithm (CS), firefly algorithm (FA), grey wolf optimization algorithm (GWA), and moth flame optimization algorithm (MFO). Automating the process of test data generation with these excellent achievements has been a burgeoning interest in recent years. Researchers [4, 5, 10] conducted a series of extensive surveys of search and found that some of these meta heuristic algorithms are widely used in the automatic software test data generation, while some have not been exploited by the test data generation techniques. Khari et al. [2] selected some algorithms according to their popularity in their research and compared the performance of the HCA, PSO, FA, CS, BA, and ABC for path coverage and branch coverage optimization. Among all, the firefly algorithm has its unique ability of automatic division and dealing with multi modal functions. It has received extensive attention and been widely used to solve optimization problems because of less parameters and simple implement.

Researchers have improved standard FA in many different ways, such as parameter control strategy, attractive model, and hybrid improvement strategy [11]. Many FA variants have been developed to solve various optimization problems. Zhao et al. [10] proposed a firefly algorithm using deep learning strategy to overcome premature convergence of the firefly algorithm. Experiments of 12 functions demonstrate its better performance. Hu [12] discussed the firefly algorithm with Gaussian disturbance which is added to the position of fireflies during iteration. Huanget al. [13] gave an improved chaotic firefly algorithm to enhance the local search ability. The Chebyshev chaotic mapping function with search operator was introduced to initialize firefly population and promote optimization during evolution process to change search area. Based on the initialized mate list and historical movement of fireflies, Waledd et al. [14] proposed a firefly photinus algorithm to change absorption parameters during optimization process to balance exploration and exploitation. Wang et al. [15] designed independent movement equations for male fireflies and female fireflies, implementing global search and local search separately. Additionally, Xie et al. [8] developed a hybrid multiobjective firefly algorithm to cope with the emerging complicated multiobjective optimization problem. Fireflies were guided by the external archive whose diversity was maintained by the archive pruning.

Also, there are some exciting achievements in software testing. Ma et al. [16] added dynamic inertia weight and compression factor to the firefly algorithm and applied it to the typical triangle type program. Transforming the test suite reduction problem into a optimization problem, Gong et al. [17] employed the firefly algorithm and greedy algorithm to obtain best solutions and then proved its reduction ability and stability. Considering the firefly movement as GA's genetic operation, Li et al. [18] combined GA with FA to reduce redundant test cases and enhance the astringency of algorithm. Pandey et al. [19, 20] developed a hybrid firefly and a genetic algorithm for regression testing environment selection and test data generation. Evaluation showed that the hybrid approach performs well.

## 3. Firefly-Based Test Case Generation

### 3.1. Test Case Generation Framework

The automatic test data generation based on FA needs to solve the cooperative operation problem between the firefly algorithm and the test date generation [21], as shown in Figure 1. The framework can be divided into two aspects: firefly algorithm and test date generation. Through close cooperation and immediate feedback, both sides promote the whole optimization process. The overall is described as follows. First, static analysis of the program under test (PUT) is performed to extract the relevant interface information. And stubs are inserted into PUT for constructing or calculating problem-specific fitness function. Next, the firefly population is initialized to the input space of PUT, where positions are decoded as parameter value. Following the principle of “moving towards brighter fireflies,” the positions of fireflies are updated in each dimension at each iteration. During the evolution process, fitness function value and coverage information are collected to further guide the optimization based on knowledge and historical experience. Evolution continues until the target solutions are found or the maximum number of generations is reached.

### 3.2. Fitness Function

In order to adapt FA to software testing area, the automatic test data generation should be converted into optimization problem, and solutions manipulated in search space should be encoded by reasonable fitness function. The encoding mechanism should ensure that neighbour solutions in search space are similar candidate test data in software testing. Better candidate solutions reflected by brighter fireflies should be rewarded, and worse candidate solutions should be punished with fitness function value. Therefore, a good fitness function is a critical factor for the efficiency and success of optimization. For test data generation, the better fitness function value should be returned for those test data which nearly meet the covering criteria.

For the automatic structural test data generation, the objective is to search test data to maximize path coverage. During the search process, we need to get feedback from execution to iterate. We focus on how far is the actual execution path for given input vector *x* away from the target path. Branch coverage is the widely used criteria in software testing [22]. Based on research achievement of Korel and Tracy [23, 24], the summation of branch function is used for structural test data generation. The fitness function for typical branch predicates can be calculated as follows (Table 1), where *k* is a constant greater than 0. By using the given fitness function, the firefly algorithm can be adapted to generate test data and then optimization process can be guided to seek better solutions.

Assuming PUT has *n* input parameters, represented as *x*_*i*_=(*x*_*i*1_, *x*_*i*2_,…, *x*_*in*_), and selected target path under test has *m* branches. Therefore, fitness function value for branch 1 is *f*_1_=*f*_1_(*x*_*i*_) and *f*_*m*_=*f*_*m*_(*x*_*i*_) for branch *m*. By summing up function value, each fitness function value for input *x*_*i*_ can be calculated as in (6), where each item is defined as in (7).

(6) $$\begin{array}{c} F=F\left(f_{1}\right)+F\left(f_{2}\right)+\cdots +F\left(f_{m}\right), \end{array}$$

(7) $$\begin{array}{c} F\left(f_{i}\right)=\left\{\begin{array}{cc} 0, & f_{i}\leq 0,\\ f_{i}, & f_{i}\geq 0. \end{array}\right. \end{array}$$

## 4. Improved Firefly Algorithm with Deep Learning

### 4.1. Motivation

In nature, the flashing fireflies are a wonderful sight especially in the summer night, and rhythmic flashing light produced by fireflies is used to attract suitable mating partners or potential prey [25]. Male fireflies have wings, so they can cruise through the air to look for favorite females While female fireflies of some species have no wings, so they usually perch on branches or grasses to wait suitable male fireflies. Once they spot a right male, they will respond to the unique pattern of flashing.

Inspired by the interesting bioluminescence character, the gender-based firefly algorithm with deep learning is proposed to accelerate the evolution in this paper. Initially, firefly population is divided into male subgroup and female subgroup, half to half. Following the mating flashing pattern, fireflies will be attracted by flashes produced by mating partners and then moved towards the brighter suitable mate. To balance the exploration and exploitation of algorithm, the movement mechanism and update formulation are designed for male and female firefly separately. Representing the global optimization ability of algorithm, male fireflies search the whole space as much as possible while female fireflies exploit local search space to find potential solutions to improve the accuracy of algorithm. Generally, the search process is promoted by excellent solutions in various nature-inspired optimization algorithms. Deep learning of excellent solutions is employed to enhance the guiding ability. Furthermore, chaotic search will be conducted near the best solution to improve the diversity and accuracy of solutions.

### 4.2. Random Attraction Model

In the standard firefly algorithm, each firefly will be attracted and moved towards any other brighter firefly, called fully attracted model [26]. Too much attraction will cause premature convergence, in which all fireflies are similar in the swarm. As a result, the convergence rate is slow and target solutions are hard to seek. Assuming there are *N* fireflies, the average movement number of each firefly is (*N* − 1)/2 [27] in each iteration and (*N∗*(*N* − 1)/2) for all fireflies. Although the fully attracted model provides a lot of opportunities for seeking, it increases the time complexity and results in oscillation, consuming considerable computing resources.

In the Gen-DLFA, male fireflies fly over the whole search space to find flashes fireflies. By adapting the randomly attracted model proposed by Wang, the male fireflies can be attracted by another randomly selected female firefly to focus on global search. Then, the max movement number of male subgroup in each iteration is (*N* − 1)/2. Comparing with the fully attracted model, the randomly attracted model has lower time complexity and reduces the attraction frequency and computing resources.

The update formula of male fireflies is defined as follows:

(8) $$\begin{array}{c} x_{i}^{t+1}=x_{i}^{t}+d\beta \lambda \left(y_{k}^{t}-x_{i}^{t}\right), \end{array}$$

where *y*_*k*_ is a randomly selected female firefly and *d* is discriminant factor of flying direction. The value of *d* is assigned based on brightness comparison. If the female firefly is brighter, *d* is set to 1; otherwise, it will be set to −1. *β* is the attractiveness between firefly *x*_*i*_ and firefly *y*_*k*_. *λ* is a random number between 0 and 1.

### 4.3. Deep Learning

In nature, the flashing light of fireflies serves as a communication mechanism to attract mating partners. According to the movement equation defined by standard FA, a firefly will be attracted and moved to any other more attractive (brighter) firefly in search space. In short, all fireflies in swarm learn from “leader.” Tang et al. [28] analyzed the trajectory of particles and employed general center particle (GCP) as learning leader in each iteration. Experiments showed that the proposed GCP can guide the evolution efficiently and improve converging speed without increasing computing complexity. The position of GCP is calculated as follows:

(9) $$\begin{array}{c} x_{d}^{\mathrm{GCP}}=\frac{1}{N}\sum_{i=1}^{D}x_{id}^{p\mathrm{best}}, \end{array}$$

where *x*_*d*_^GCP^ is the *d*th spatial coordinate of general center particle and *x*_*id*_^*p*best^ is the *d*th spatial coordinate from memory of particle *i*.

Benefit from excellent leadership of GCP in SPO, the general center of male fireflies can be constructed by historical best values from their leaning memory to attract female fireflies. As other fireflies, the general center firefly can emit flashing light to participate in cooperative communication and guide the search process of female fireflies with its leadership strength.

In order to discover useful patterns and intrinsic feature of training data from experience, the deep learning technique builds complex mapping relationship between low level features to high level semantics of training data. Hu et al. [29] adopted the deep neural network to recognize faults in bogies. Wang et al. [30] proposed an attention-based deep learning framework for trip destination prediction. Chen et al. [31] proposed an improved semantic segmentation neural network, which adopted a fully connected (FC) fusion path and pretrained encoder for the semantic segmentation task of HRRS imagery. Inspired by these exciting achievement, deep learning is employed on general center firefly to promote its leadership advantage during evolution process, enhancing the global search ability.

Initially, the general center firefly is used as input for the deep learning model. Then, the single dimension optimization is carried out with count times according to the following equation:

(10) $$\begin{array}{c} x_{d}^{\mathrm{GCP}}\left(t+1\right)=x_{d}^{\mathrm{GCP}}\left(t\right)+\mathrm{cauchy}\left(\right)\left(x_{rd}\left(t\right)-x_{d}^{\mathrm{GCP}}\left(t\right)\right), \end{array}$$

where *x*_*rd*_(*t*) is the *d*th spatial coordinate of the randomly selected firefly *r* and *x*_*d*_^GCP^(*t*) is the *d*th spatial coordinate of general center firefly at the *t*th iteration.

The general center firefly generated from deep learning architecture is used to guide the evolution process of female fireflies to learn from historical experiments. If the general center firefly is brighter than female one, the female firefly should move and update its position according to (11); otherwise, female firefly mutates according to (12).

(11) $$\begin{array}{c} x_{id}\left(t+1\right)=x_{id}\left(t\right)+\beta_{0}e^{-\gamma r_{i\mathrm{GCP}}^{2}}\left(x_{d}^{\mathrm{GCP}}\left(t\right)-x_{id}\left(t\right)\right), \end{array}$$

(12) $$\begin{array}{c} x_{id}\left(t+1\right)=x_{d}^{g\mathrm{best}}\left(t\right)+\text{cauchy}\left(\;\right), \end{array}$$

where cauchy() is random number generated by Cauchy distribution function and *x*_*d*_^*g*best^(*t*) is the *d*th spatial coordinate of the brightest firefly in the search space at iteration *t*.

### 4.4. Chaotic Search

Ideally, fireflies will slowly gather together and then focus on the best solutions at the end. However, at the final period of searching, distance between any other fireflies decreases, thus increasing the attractiveness. Too much attraction increases the movement, and it is difficult to find target solutions because of oscillation caused by too much movement.

Like other well-known global optimization methods, the firefly algorithm should balance the intensification and diversification. Recently, chaos has drawn more attention in various applications, including optimization algorithms, data encryption, and smartphone fitting algorithm [32]. Gandomi et al. [33] introduced 12 different chaotic maps into FA and proved its improved global search ability for robust global optimization. After position update of all fireflies, chaos search is employed to seek around the current global best solution *x*^*g*best^ to improve seeking accuracy. During the chaotic search process, chaotic variables generated by chaotic sequence are mapped into input space initially. Then, some candidate solutions will be selected due to ergodicity and disturbance properties of chaos. The chaos strategy can effectively overcome the typical local optimal problem and explore search space of standard FA. The detailed steps can be described as follows:

Firstly, chaotic sequence generated by logistic mapping function is represented as follows:
  (13) $$\begin{array}{c} ch_{0}=\mathrm{rand}\left(\right)\\ ch_{k+1}=\alpha *ch_{k}\left(1-ch_{k}\right), \end{array}$$
where *ch*0 is the initialized random number between 0 and 1, *k* is the iteration number, and *ch*_*k*_ is the *k*th number in chaotic sequence. Obviously, all chaotic number will between 0 and 1 under the initial condition of *ch*0. *α* is set 4, and *k* is set 5 to ensure the completeness of search space.
Secondly, chaotic sequence is mapped to search space as follows:
  (14) $$\begin{array}{c} Ch_{k}=L+ch_{k}*\left(U-L\right), \end{array}$$
where *ch*_*k*_ is the *k*th chaotic number in sequence and *U* and *L* are upper bound and lower bound of parameters of programs under test.
Finally, chaotic search is conducted near the best solution *X*^*g*best^ according to (15) to obtain *k* solutions to enhance the local exploitation ability and improve the search precision:

(15) $$\begin{array}{c} \varepsilon =\frac{\mathrm{ItMax}-t+1}{\mathrm{ItMax}}\\ x^{g\mathrm{bes}t^{\prime }}=\left(1-\varepsilon \right)x^{g\mathrm{best}}+\varepsilon *Ch\left(k\right). \end{array}$$

### 4.5. Proposed Algorithm of Gen-DLFA

The process detail of Gen-DLFA is described as follows:

1. Firefly population and relative parameters are initialized, and then the population is divided into male group and female group;
2. Each male firefly will randomly select another female firefly and update its position in each dimension according equation (8);
3. General center firefly of male group is constructed from their historical experiment by equation (9). Then, conduct deep learning count times by equation (10);
4. The general center firefly will guide the optimization process of female subgroup. If the general center firefly is brighter than female one, the female firefly should move and update its position in each dimension according equation (11); otherwise, female fireflies mutate according to equation (12);
5. Chaos search is implemented around the current best solutions to generate *k* candidate solutions by equation (15) to improve accuracy and population diversity;
6. It is checked whether the stopping condition is satisfied. If the conditions are met, the search process stops and outputs the best solutions. Otherwise, the search process goes back to step 3.

Based on above analysis, the pseudo code of the gender difference-based firefly algorithm with deep learning (Gen-DLFA) can be summarized in Algorithm 1. Some key parameters are defined as follows: maxGen is the max generations of evolutions, *N* is the population size, and *g*best represents the global best firefly at each generation.

## 5. Empirical Evaluation

The goal of the experiment is to evaluate performance of Gen-DLFA. Some benchmark programs and state-of-the-art firefly algorithm variants are used to conduct comparison analysis. Specially, we investigated the following research questions:

 
*RQ1 (Effectiveness).* Whether Gen-DLFA can seek target solutions for structural test case generation? What is the average coverage rate? Does it perform better?
 
*RQ2 (Efficiency)*. What is the rate of convergence? How much computing resource will be required for target solutions? What extent of cost can the Gen-DLFA reduce?
 
*RQ3 (Diversity).* How many different target solutions found during the total optimization process?

### 5.1. Experiment Preparation

#### 5.1.1. Test Objects

Some benchmark programs which were widely used in software test data generation were selected to assess the performance of Gen-DLFA [20, 34].  Table 2 shows the details of the programs under test. Although the scale of programs is limited, their input space dimensions vary from 2 to 8 and so on. The branch number of each program under test ranges from 5 to 36. As seen from table, the target branches are the deep nested paths with strict conditions, which represent the objectives to be optimized. With respect to the searching difficulty, these optimization targets ensure the diversity and complexity of experiments.

#### 5.1.2. Experimental Setup

We carried out an empirical study to assess the Gen-DLFA with standard FA and three other FA variants. Parameters of each algorithm are shown in Table 3. For the sake of fairness, the population size of all algorithms was chosen to be 100 and the maximum generation number was set to 7000. Additionally, each experiment was repeated 30 times independently and the average value of experimental results was used to reduce deviation caused by randomness. The input data of PUT were encoded as firefly position, while the number and bounds of parameters of PUT define the whole input space. All benchmark programs used for comparative experiments were written in Java, and most of them can be found in source code lib of Liang [35]. The experiments were performed under the common testing environment: win 10 pro 64 bit operating system, Java Se development kit 9, Intellij IDEA, Intel Core i7 processor, and 8 GB, LPDDR3 memory.

### 5.2. Effectiveness

The success coverage rate is used to measure the effectiveness of algorithms in this paper. For signal target path coverage, it can be calculated as the number of success search divided by the total times of search. In our experiments, coverage means how many times the algorithms can find target solutions satisfying the selected branch covering criterion over repeated 30 independent implementations. The coverage results are summarized in Table 4.

As seen from Table 4, the overall average coverage for FA and Gen-DLFA is 95%. Each firefly is attracted and moved towards any other brighter firefly in FA. This fully attracted model gives fireflies more learning opportunities, which ensure the sufficiency of optimization. The overall average coverage for RaFA is 74%, in which each firefly is attracted by the randomly selected firefly to reduce the attraction frequency and then accelerate the evolution process. Although RaFA is easier to implement, its global search ability and search precision are relatively weak. The rate is not stable for each program, varying from 30% to 100%. The average rate of other algorithms is similar, 80% for DLFA and 83% for GDFA, employing deep learning strategy and gender subgroups separately. Gen-DLFA outperforms better than other four algorithms except for the program LineCover, which requires high precision than others.

### 5.3. Efficiency

The consumption of search budget is used to measure the efficiency of algorithms for comparative analysis. For automated structural test case generation, we use the average convergence generations and the average search time (measured in ms) as measure metrics. That is, we focused on overall average generations and average optimization time consumed by successful search, which can seek target solutions that satisfied the selected coverage criterion.  Table 5 presents the experiment results.

In order to compare the search consumption of multiple algorithms on benchmark programs, we calculated the total average value at the last row in Table 5, indicating average convergence generations and run time, respectively. From the results, we can see that the standard FA finds reasonable solutions with the least average generations 1710. However, it consumes the most 40453 ms run time among all algorithms because of lots of attractions caused by the fully attracted model. Compared with the standard FA, RaFA takes much less time but more generations to seek the target solutions. Its total average convergence generations are 2335 while the average run time is 3475 ms. The performance is not stable since the dependence on the randomized initialization of population in some extent. With 2178 average generations and 17853 ms run time, the performance of proposed Gen-DLFA is similar to that of DLFA and better than that of GDFA in general.

As a typical benchmark program, the source code of triangle has been widely used in the research of automatic test data generation. Its average convergence generations and run time for equilateral triangle are import performance measures for evaluating various algorithms. As seen from Table 4, the standard FA spent 22909 ms on searching target solutions through 1468 times generations, the most computation resource consumption among all algorithms. Notably, the Gen-DLFA found the best solution with 1023 generations in 6210 ms, achieving promising results at a lower search cost. It shows more robust performance than other algorithms on most benchmark programs.

### 5.4. Stability

In order to verify the performance of algorithms, some additional experiments were conducted for discussing the implementation detail to check the stability and observing the performance volatility with the population size.

As for the performance of each algorithm in different experiments, several programs are selected from Table 2. Once the ranges of input parameters for each program were defined, they kept the same value during the whole execution. The result of convergence generation for each algorithm collected from 30 times execution is shown in Figure 2. As seen, the average convergence generations of Gen-DLFA for triangle, RectOverlap, and LineRect are lower than those of other algorithms. While for Quadratic, the average convergence generations of Gen-DLFA and FA are similar but lower than those of DLFA and GDFA. In addition, the convergence generations of Gen-DLFA are stable with little fluctuation.

The population size is one of the key factors to algorithm performance. Taking the triangle program, for example, the convergence generations under different population size are shown in Figure 3. It can be seen from the figure that the average convergence generation decreases with the increment of population size and tends to stable when reaching a certain population size. In most cases, Gen-DLFA and FA can find the target solutions with less convergence generations.

### 5.5. Diversity

The positive feedback strategy adopted by many metaheuristic algorithms can accelerate the convergence rate but may result in population premature and low population diversity. Researchers have proposed various approaches to keep a balance between diversity and convergence. The better diversity of solutions, the stronger ability of test cases to detect defects in software testing.

For simplicity, we use the different solutions rate to measure diversity, which can be calculated as the solutions with different values divided by the total success research. Taking the typical benchmark program triangle, for example, the detailed diversity rate of all algorithms is summarized in Figure 2. To obtain a fair analysis, all algorithms use the same settings. Each algorithm runs independently many times to get 20 target solutions. As seen from Figure 4, the standard FA and its variants perform well. The diversity of all algorithms improves with the increment of parameters' input space. Gen-DLFA shows better performance and achieves promising results.

## 6. Conclusions

Generally, software test data generation is extremely laborious and costly for software engineers in industry. As an extremely active branch of search-based software engineering, some typical metaheuristic algorithms and their variants have been proved to be an effective way of generating realistic test data. Aiming at some drawback of the firefly algorithm, such as premature convergence and low search accuracy, we proposed the gender-based firefly algorithm with deep learning (Gen-DLFA) to generate realistic structural test data. Initially, the population was divided into male subgroup and female subgroup. Employing the randomly attracted model, each male firefly is attracted by another randomly selected female firefly, representing the global search ability, while female fireflies implement local search guided by the general center firefly constructed through certain times of one-dimensional deep learning. Thus, Gen-DLFA can balance the exploration and exploitation well. Furthermore, the chaotic search is conducted near the best solution in Gen-DLFA to improve the diversity and accuracy of solutions. The comparison results indicate that Gen-DLFA can achieve better performance in terms of effectiveness, efficiency, and diversity. The proposed algorithm showed a strong search ability and found target solutions at a reasonable computational cost.

As further research, more studies are needed in the controlling parameters setting, population diversity maintenance, stability of the firefly algorithm, and so on. In addition, most of the research studies have focused on single objective optimization, and it will be useful to focus on multiobjective optimization incorporating with current metaheuristic algorithms.

## Figures and Tables

**Figure 1:** Test data generation workflow.

**Figure 2:** Distribution of average convergence generations: (a) triangle; (b) RectOverlap; (c) Quadratic; (d) LineRect.

**Figure 3:** Population size vs. convergence generation.

**Figure 4:** Diversity analysis.

**Algorithm 1:** The pseudo code of Gen-DLFA.

**Table 1:** Branch distance for several predicates.

Predicates	Branch distance function
Boolean	If true, then 0; else *k*
¬*a*	Negation is propagated over *a*
*a* = *b*	If *abs*(*a* − *b*)=0, then 0; else (*a* − *b*)+*k*
*a* ≠ *b*	If *abs*(*a* − *b*) ≠ 0, then 0; else *k*
*a* < *b*	If *a* − *b* < 0, then 0; else (*a* − *b*)+*k*
*a* ≤ *b*	If *a* − *b* ≤ 0, then 0; else (*a* − *b*)+*k*
*a* > *b*	If *b* − *a* < 0, then 0; else (*b* − *a*)+*k*
*a* ≥ *b*	If *b* − *a* ≤ 0, then 0; else (*b* − *a*)+*k*
*a* and *b*	*f*(*a*)+*f*(*b*)
*a* or *b*	min(*f*(*a*), *f*(*b*))

**Table 2:** Benchmark programs under test.

Programs	Parameters	Target branch	Description
Triangle	*x*, *y*, *z*	(*x* = = *y*) && (*y* = = *z*) is true (equilateral triangle)	Calculates whether a triangle defined by inputs *x*, y, and *z* is equilateral, isosceles, or scalene.
Angled	*x*, *y*, *z*	*x* ^2^ + *y*^2^ − z^2^ = = 0 is true	Check whether the given inputs *x*, *y*, and *z* satisfy the criteria of right triangle.
RectOverlap	*x*1, *y*1, *w*1, *h*1, *x*2, *y*2, *w*2, *h*2	Two rectangles overlap	Check relationship between two rectangles represented as *x*1, *y*1, *w*1, *h*1, *x*2, *y*2, *w*2, and *h*2.
Quadratic	*a*, *b*, *c*	*b∗b* − 4*∗a∗c*==0 is true	Judge the roots type of the quadratic equation with one variable (*ax*^2^ + *bx* + *c* = 0).
Nextday	year, month, day	Next day is Feb. 28^th^ in leap year	Calculate next day of the given input year, month, and day.
LineCover	*x*1, *y*1, *x*2, *y*2, *x*, *y*, *w*, *h*	A line segment is the diagonal of a rectangle	Check whether a line defined by (*x*1, *y*1) and (*x*2, *y*2) is the diagonal of a rectangle. (*x*, *y*) is the coordinates of lower left point of the rectangle.
LineCircle	*x*1, *y*1, *x*2, *y*2, *x*, *y*, *r*	A line segment is tangent to a circle	Calculate relationship between a line segment and a circle. (*x*1, *y*1), (*x*2, *y*2), and (*x*, *y*) are coordinates of a line and a circle.
LineRect	*x*1, *y*1, *x*2, *y*2, *x*, *y*, *w*, *h*	A line segment intersects at a rectangle	Calculate the position relationship between a line segment and a rectangle. It can be divided into inclusion, intersection, and disjoint.

**Table 3:** Algorithms for experimental analysis.

Algorithm	Parameters	Reference
FA	*α* = 0.2, *β*0 = 1.0, *γ* = 1.0	Yang 2010 [35]
FA with random attraction (RaFA)	*α* = 0.2, *β*0 = 1.0, *γ* = 1/Г^m^ (*m* = 2)	Wang et al. 2016 [26]
Deep learning FA (DLFA)	*α* = 0.2, *β*0 = 1.0, *γ* = 1/Г^m^ (*m* = 2)	Zhao Jia et al. 2018 [9]
FA based on gender difference (GDFA)	*β*0 changed with functions under test and	Wang et al. 2019 [15]
Gen-DLFA	*α* = 0.2, *β*0 = 1.0, *γ* = 1.0	N/A

**Table 4:** Success coverage rate.

Programs	FA	RaFA	DLFA	GDFA	Gen-DLFA
Triangle	100	42	90	62	100
Angled	100	95	65	70	100
RectOverlap	100	100	73	82	100
Quadratic	100	100	70	90	100
Nextday	100	30	85	100	100
LineCover	70	64	77	90	60
LineCircle	92	58	78	74	100
LineRect	100	100	100	100	100
Avg.	95	74	80	83	95

**Table 5:** Average convergence generations and search time.

Programs	FA	RaFA	DLFA	GDFA	Gen-DLFA
Triangle	1468/22909	4293/4258	2219/7317	2099/13633	1023/6210
Angled	2123/28272	2615/3793	5183/20347	4784/13356	4120/18580
RectOverlap	828/15637	1919/2947	844/8935	2826/11414	593/7362
Quadratic	908/15054	1317/2648	2340/9786	2864/17584	1203/7958
Nextday	1190/2018	333/339	446/1302	1870/5066	1325/1915
LineCover	2623/57493	2274/3913	6783/28444	3450/17402	4939/21976
LineCircle	3196/174268	4897/8668	5368/93477	6290/92304	4012/74695
LineRect	424/7980	1030/1238	840/6382	284/6708	214/4135
Avg	1710/40453	2335/3475	3002/21998	3058/22183	2178/17853

## Data Availability

The research related data consists of two parts: pseudocode of the proposed algorithm and its corresponding benchmark programs under test. The pseudocode of Gen-DLFA data to support the findings of this study (detailed in Algorithm 1) and the benchmark programs under test data are included within the article (detailed in Table 2).
